RETRACTED

# Microbiome restoration diet improves digestion, cognition and physical and emotional wellbeing

**DOI:** 10.1371/journal.pone.0179017

**Published:** 2017-06-14

**Authors:** Kate Lawrence, Jeannette Hyde

**Affiliations:** 1 Department of Psychology, St Mary’s University, Twickenham, United Kingdom; 2 Independent researcher, registered nutritional therapist BSc (Hons) Nutritional Therapy CNHC mBANT, Twickenham, United Kingdom; University of Palermo, ITALY

## Abstract

Manipulating gut bacteria in the microbiome, through the use of probiotics and prebiotics, has been found to have an influence on both physical and emotional wellbeing. This study uses a dietary manipulation ‘*The Gut Makeover*’ designed to elicit positive changes to the gut bacteria within the microbiome. 21 healthy participants undertook ‘*The Gut Makeover*’ for a four week period. Weight and various aspects of health were assessed pre and post intervention using the Functional Medicine Medical Symptoms Questionnaire (MSQ). Paired sample t-tests revealed a significant reduction in self-reported weight at the end of the intervention. Adverse medical symptoms related to digestion, cognition and physical and emotional wellbeing, were also significantly reduced during the course of the dietary intervention. The intervention, designed to manipulate gut bacteria, had a significant impact on digestion, reducing IBS type symptoms in this non-clinical population. There was also a striking reduction in negative symptoms related to cognition, memory and emotional wellbeing, including symptoms of anxiety and depression. Dietary gut microbiome manipulations may have the power to exert positive physical and psychological health benefits, of a similar nature to those reported in studies using pre and probiotics. The small sample size and lack of control over confounding variables means that it will be important to replicate these findings in larger-scale controlled, prospective, clinical trials. This dietary microbiome intervention has the potential to improve physical and emotional wellbeing in the general population but also to be investigated as a treatment option for individuals with conditions as diverse as IBS, anxiety, depression and Alzheimer’s disease.

## Introduction

The intestines of an average human contain trillions of gut bacteria. The diversity and strains of these bacteria vary dramatically between individuals. Research has shown that sub-optimal gut bacteria can have a profound impact on health. For example, the health of the microbiome, in terms of species and diversity of gut bacteria, has been found to be associated with digestive issues, such as nausea, bloating and diarrhoea [1] and Irritable Bowel Syndrome (IBS) [2]. Additionally, sub-optimal bacterial diversity is reported in a number of conditions that have a severe impact on health, from Crohn’s disease [3], and obesity [4] to type 2 diabetes [5].

RETRACTED

The ecology of the gut microbiome has been connected with weight in animal studies [6, 7]. Low bacterial richness has been linked with higher body mass index in humans, and bacterial richness with lower body mass index [8]. Low diversity of fecal bacteria was recently connected specifically with visceral fat in human twin studies [9]; with visceral fat being linked with a higher risk of cardiovascular disease and type 2 diabetes [10].

Gut bacteria have been hypothesized to influence weight by signalling satiety to the brain in animal studies [11] and by influencing caloric extraction from food [12]. The microbiota of obese youths have, for example, been shown to be more efficient at oxidising carbohydrates into storable fat than those of lean youths [13]. Additionally, evidence from murine studies suggests that, bacterial diversity plays a role in host metabolism and obesity [14].

Some studies have explored the influence of orally administered probiotics on weight in both human and animal populations. Probiotics consist of a range of micro-organisms (i.e. beneficial bacteria) that are introduced into the body with the view of gaining a health benefit from them [15]. The Lactobacillus genus of bacteria, in particular, would appear to play a role in weight regulation [12] perhaps mediated by its involvement in the fermentation of sugars into acids [16].

Despite some inconsistency in study findings, orally administered probiotics have also been reported to help alleviate gastrointestinal symptoms in IBS [17,18]. However, as yet, it is unclear whether beneficial probiotic effects (especially in healthy adults) are mediated by directly altering the state of our gut microbiota [19], [20]. More research is needed to discover whether probiotic supplementation can have health benefits for non-clinical populations.

Taking oral probiotics, as a supplement, is not the only means by which we can influence our microbiome. The make-up of our gut bacteria does not necessarily remain stable throughout life [21] and can be influenced by factors such as parasites, disease and our environment [22, 23]. Diet can rapidly influence the richness of bacteria in the gut with consequences for health [24] and is the most important influence on the microbiome [25]. Research has shown that gut bacteria can be manipulated in a matter of days by alterations to diet. For example, altering the amount of vegetable-based or animal-based food within the diet, as well as adjusting carbohydrate intake, can influence the make-up of the microbiome [26,27]. A four-week gut bacteria restoration program *The Gut Makeover*’ is a dietary protocol which attempts to manipulate gut bacteria by restricting processed high grain carbohydrate foods, sugar, and artificial sweeteners, which may cause dysbiosis, together with increasing the consumption of vegetables and fermented foods which promote beneficial bacteria [28]. This diet was devised primarily as a tool for weight-loss and resolution of digestive symptoms. However, anecdotal reports of people taking part in this program suggest supplementary improvements in both physical and psychological wellbeing [28].

RETRACTED

Although the effect of *The Gut Makeover* diet on the health and diversity of the microbiome has not been directly tested, its conceptualisation was based upon science that suggests these manipulations would promote gut health and a diverse microbiome. Recommendations include consuming a wide variety of vegetables and fruit containing fibre [29,30] and phytochemicals [30] to feed gut bacteria and promote diversity of species. Individuals are encouraged to eat probiotic foods, to plant beneficial bacteria in the gut [31], and prebiotic foods, to feed gut bacteria [24,32]. Time restricted feeding is also suggested, which involves fasting for twelve hours between dinner and breakfast, to allow the gut time to stimulate gut bacteria regrowth overnight [14,33].

Previous research has identified significant reductions in adverse digestive symptoms [17] and improvements in weight regulation [12], mood [34] and other aspects of general health and well-being [35] for individuals who take probiotics. In this exploratory study, we investigated whether a dietary intervention, designed to manipulate gut bacteria, could have a positive effect on physical and emotional well-being in healthy adults.

## Materials and methods

This retrospective assessment of nutritional therapy work (with no control group) was based on a repeated-measures design. Participants had all undertaken group nutritional therapy as part of routine clinical practice. St Mary’s University Ethics Committee granted ethical approval for the researchers to contact the participants taking part in this therapy to request permission to use their data for a research study. All except two participants consented; one was non-contactable and the other did not wish for their data to be used. All participants gave written informed consent for their before and after data to be used for research purposes. The study was carried out on 21 participants (20 females and 1 male) aged 27 to 64 years, mean age 47 years. Of the participants, 20 were Caucasian and one Asian.

RETRACTED

As a part of routine group nutritional therapy, participants had followed the dietary program (designed to optimise gut bacteria) for 4 weeks, completing a questionnaire about their health and well-being before the diet and after the diet.

### Dietary program to optimise gut bacteria

*The Gut Makeover* [28], is a dietary program that was designed to improve the health and diversity of the microbiome, leading to weight loss and subsidiary health benefits (primarily digestive). The groups were a convenience sample of people seeking the services of a nutritional therapist. The majority of participants’ primary goal was therefore weight-loss, with several additionally aiming to improve digestive symptoms (chronic acid reflux, bloating, constipation, loose stools, wind), plus energy, and pain issues. None of the participants took part in the nutritional therapy with the explicit aim of improving emotional or cognitive well-being.

Participants either attended an in-person or online workshop at the start of the program, where they were briefed by a nutritional therapist, trained in the procedure, on the dietary protocol for the four-weeks. They were also given handouts detailing the plan. Further in-person or online conference call group briefings with the nutritional therapist were conducted at the half-way point of the diet (after two weeks) and at the end (after four weeks). A private Facebook group was also offered to both groups during the program where they could share experiences and ask the nutritional therapist questions.

*The Gut Makeover* protocol was developed based on research into the microbiome and gut permeability. Details of the protocol are described fully in the published guidelines [28] and summarised below.

#### Throughout the four weeks, participants

- Eat three main meals per day, no snacks between.
- Undergo a 12-hour overnight fast between dinner and breakfast, with just water permitted between.
- Eat seven American cupfuls of plants (uncooked volume) per day (five as vegetables, two as fruit).
- Eat protein with each meal (either animal, fish, eggs, nuts, or seeds).
- Eat between 20 and 30 different types of plants (fresh herbs, vegetables, and fruits) over the course of a week for variety.
- Use extra virgin olive oil and coconut oil as their default cooking oils.
- Chew food thoroughly–aiming for approximately 20 chews per mouthful.
- Do not count or restrict calories.

#### In the second half of the plan (weeks 2–4) participants also

- Can eat butter and ghee.
- Consume probiotic foods such as fermented milk kefir, sauerkraut, tempeh, and miso.
- Increase their intake of prebiotic vegetables such as bananas, fennel, asparagus, cold potatoes, onions, garlic, leeks, fennel, Jerusalem artichokes, pak choi.
- Consume bone broth/stock.

RETRACTED

#### Excluded from the diet throughout the four weeks

- Refined sugars.
- Grains (e.g. wheat, rice, oats, maize, quinoa) and pulses (e.g. lentils and beans)
- Alcohol
- Caffeine
- Dairy (can be reintroduced after 2 weeks if no adverse symptoms on re-introduction)

The research aimed to quantitatively assess the impact of *The Gut Makeover* program on different aspects of health and wellbeing. This was assessed using the Functional Medicine Medical Symptoms Questionnaire (MSQ) [36], which consists of 71 questions, relating to 15 areas of health (detailed in Table 1), including symptoms related to the digestive tract, the mind and emotions. The MSQ [36] is a tracking tool used by clinicians to assess patient progress to dietary and lifestyle changes. It was given to participants, as part of their routine intervention, to assess any changes in symptoms from pre- to post-intervention. It was not selected specifically for the purpose of research, and is lacking in detailed information relating to its reliability and validity compared to scales used more specifically for research. Nonetheless, it contains valuable information which can be explored to guide further hypothesis-driven research. A Cronbach’s alpha test, conducted on our pre-assessment responses, revealed an α value of .926, indicating excellent internal consistency of the MSQ. Post-intervention responses to the scale items also indicated a high level of internal consistency to the scale (α = .827).

**Table 1:** Question items and range of scores for each subscale of the Medical Symptoms Questionnaire (MSQ).

Subscale	Number of items	Example symptom	Potential range of scores
**Head**	4	Dizziness	0–16
**Eyes**	4	Watery or itchy eyes	0–16
**Ears**	4	Ear aches, ear infections	0–16
**Nose**	5	Sneezing attacks	0–20
**Mouth/throat**	5	Canker sores	0–20
**Skin**	5	Acne	0–20
**Heart**	3	Rapid or pounding heartbeat	0–15
**Lungs**	4	Shortness of breath	0–16
**Digestive tract**	7	Diarrhea	0–28
**Joints/muscle**	5	Pain or aches in joints	0–20
**Weight**	6	Binge eating/drinking	0–24
**Energy/activity**	4	Fatigue/sluggishness	0–16
**Mind**	8	Poor concentration	0–32
**Emotions**	4	Anxiety, fear, nervousness	0–16
**Other**	3	Frequent or urgent urination	0–12
**Total**	71		0–284

Participants were requested to rate each of the following symptoms based upon their typical health profile for the past 14 days and responded to each item on a five point scale, ranging from 0–4, to indicate the presence or absence of each symptom. Zero indicates never or almost never and mild, whilst a rating of four indicates severe and/or frequent symptoms. The subscales contain different numbers of questions and therefore different ranges of possible scores; this information is detailed in Table 1.

RETRACTED

Participants completed the questionnaire at time point one (the beginning of *The Gut Makeover* program) and at time point two (on completion of the four-week program). The questionnaire was handed to participants to complete as a paper copy within the room in which the sessions with the nutritional therapist were run or sent to participants at their home. The questionnaires took approximately 10–15 minutes to complete. Once the questionnaires were completed, they were returned to the nutritional therapist. Scores for each sub-section were totalled to give a severity of symptoms score for each health area, together with an overall score. A low score is indicative of few/mild symptoms and a high score indicative of many/more severe symptoms.

## Results

Of the 21 participants, 20 reported their weight at time point one, and time point two. Weights were self-recorded and subjects were asked to weigh themselves on the same set of scales, at the same time of day, at the start and end of the program. Weight loss ranged from 1kg (2.2 pounds) to 7kg (15.4 pounds). The mean weight loss for females was 3.2kg (7.1 pounds), SD 1.6kg (3.5 pounds) and the weight loss for the single male participant was 4.1kg (9.0 pounds) A paired sample t-test revealed a highly significant effect of the intervention, with weights being lower post-intervention (female mean 65.3kg, SD 9.78; male 95.1kg) than pre-intervention (female mean 68.5kg, SD 10.68kg; male 99.2kg) (t (21) = 9.17, p < .0001).

Within the clinician debrief, a range of gastro-intestinal improvements were reported by participants and included: reduction or cessation of chronic bloating, acid reflux, wind, erratic stool movements (either loose or constipation, or chronic alternation between the two). Also noted were self-reported improvements in mood, energy and quality of sleep.

Total medical symptoms scores were submitted to a paired-sample T-test. Total scores at time 1 (before dietary intervention) and time 2 (after the four week dietary intervention) were entered as the paired variables. There was a significant effect of dietary intervention on medical symptoms (t (21) = 7.87, p < .0001). As can be seen in Fig 1, the number and severity of medical symptoms reported before the intervention (mean = 60.10, SD = 31.95) was more than 3 times greater than that reported after the four-week dietary intervention (mean = 18.71, SD = 12.69).

**Fig 1:** Total medical symptoms score before and after four-week dietary intervention. Error bars show 95% confidence intervals.

RETRACTED

Without exception, all participants saw a drop in their total medical symptoms scores from before the intervention to post-intervention; these symptom score changes are depicted in Fig 2. No participant saw their symptom score increase, or stay the same, from pre-intervention to post-intervention.

**Fig 2:** Total medical symptoms score before and after dietary intervention for each participant.

Total scores for each of the 14 subscales of the Medical Symptoms Questionnaire (MSQ) were then entered into paired-sample t-tests. Since 14 tests were conducted, Bonferroni corrections were applied to the significance level (.05/14) re-setting it to .0036. After this correction was applied, a significant difference between symptom scores, before and after the dietary intervention, was found for 11 of the individual subscales. For all of these subscales, fewer medical symptoms were reported post-intervention (see Table 2). There was a significant effect of dietary intervention for head symptoms (t (20) = 4.95, p < .0001), eye symptoms (t (20) = 3.96, p = .001), nose symptoms (t (20) = 4.22, p < .0001), skin symptoms (t (20) = 4.78, p < .0001), heart symptoms (t (20) = 4.11, p = .001), digestive symptoms (t (20) = 6.10, p < .0001), joint and muscle symptoms (t (20) = 4.66, p < .0001), weight symptoms (t (20) = 6.47, p < .0001), energy symptoms (t (20) = 5.18, p < .0001), mind symptoms (t (20) = 5.22, p < .0001), and emotion symptoms (t (20) = 7.67, p < .0001).

**Table 2:** Pre- and post-intervention total scores for each of the subscales of the Medical Symptoms Questionnaire.

Symptom subscale	Symptoms total before intervention Mean (SD)	Symptoms total after intervention Mean (SD)	P-value
**Head**	3.43 (2.04)	1.19 (1.29)	< .0001
**Eye**	3.81 (3.11)	1.52 (1.57)	= .001
**Ear**	1.29 (1.82)	.67 (1.46)	n/s
**Nose**	4.14 (3.23)	1.29 (1.95)	< .0001
**Mouth and throat**	2.86 (3.80)	1.00 (2.00)	n/s
**Skin**	4.38 (3.63)	1.71 (2.31)	< .0001
**Heart**	1.24 (1.30)	0.14 (0.48)	= .001
**Lungs**	0.86 (1.85)	0.14 (0.48)	n/s
**Digestive**	8.57 (5.56)	2.42 (2.66)	< .0001
**Joint and Muscle**	4.95 (4.66)	2.24 (3.08)	< .0001
**Weight**	8.33 (5.76)	0.90 (1.14)	< .0001
**Energy**	4.95 (4.06)	1.33 (1.98)	< .0001
**Mind**	4.24 (3.86)	1.14 (1.74)	< .0001
**Emotion**	5.33 (3.57)	1.76 (2.00)	< .0001

## Discussion

*The Gut Makeover* program was developed with the aim of optimising the health and diversity of the microbiome and thereby promoting weight-loss and helping to resolve digestive issues. Results of this exploratory study revealed that the program did indeed produce significant reductions in self-reported weight and also in symptoms on weight subscale of the MSQ. Participant responses on the weight sub-scale of the MSQ suggest that issues such as binge eating, cravings, carrying excessive weight, compulsive eating and water-retention improved with the four-week intervention. If we assume that adherence to the diet had an influence on the health and diversity of the microbiome, this fits with research which suggests that the microbiome appears to play an important role in energy regulation [12]. Transplanting faeces from obese individuals into mice has been found to induce weight gain in the mice [37] suggesting a direct effect of microbiota in influencing weight which can occur rapidly upon microbiome modification. However, long-term maintenance of a lean phenotype, resulting from transplant, is not yet well-demonstrated and likely requires dietary modification to support the additional microbial diversity[38,39]. In humans, more diverse microbiomes are associated with lower weight and less visceral fat [8,9] and in theory *The Gut Makeover* intervention should promote greater microbiome diversity [28]. It is unknown whether calorie intake was reduced from pre-intervention levels, due to the removal of certain foods from the diet. However, the diet required no calorie or portion size restriction and allowed unrestricted use of extra virgin olive oil, butter, and coconut fat, meaning that a reduction in calorific intake was not an intended consequence of the diet.

RETRACTED

The participants, in this observational study, also saw a significant reduction in self-reported digestive symptoms on the MSQ; there was a lower frequency and severity of nausea, vomiting, diarrhoea, constipation, bloating, passing gas, heartburn and stomach pain after the four-week intervention. Our study attempted to manipulate gut bacteria, not by probiotic supplements, but through the use of diet to promote beneficial bacteria. Our findings are consistent with research suggesting that enhancing gut bacteria, through probiotic interventions, can alleviate some of the symptoms of IBS [17,18]; with the further suggestion that similar digestive improvements may be achieved through dietary therapy. Additionally, these benefits may be realised, not just in individuals with diagnosed gut conditions, but also in ‘healthy’ adults.

Improvements in weight and digestion were expected outcomes for participants undertaking this protocol. We were, however, more surprised by the positive impact of the intervention on a vast range of other areas of well-being. Head symptoms (such as headaches, faintness, dizziness and insomnia) decreased, as did symptoms related to the eyes, nose, skin, heart and joints. Participants also reported a positive impact on energy levels. Scores for symptoms related to negative emotions also fell significantly.

RETRACTED

Analysis of scores, on the ‘emotions’ sub-section of the MSQ, revealed that there was a significant improvement in emotional well-being after the four-week program. The symptom score for emotional dysfunction was three times higher before the intervention than it was after taking part in the four-week program. There was a reduction in mood swings, anxiety, irritability and depression. For participants, this was an unexpected benefit of the treatment; none of the participants had taken part in dietary regime with view to it having benefits with regard to mental-health. This means that the positive impact on emotional-wellbeing is unlikely to have been influenced significantly by participant expectations. However, since emotional wellbeing is also closely related to physical wellbeing and body image [40,41] it could be that the psychological benefits are an indirect result of microbial augmentation, mediated by weight-loss and reduction in physical ailments.

An improvement in emotional well-being is consistent with other studies which have used more direct manipulations to influence the microbiome. In mice, who have been stripped of their gut bacteria, higher levels of cortisol (the stress hormone) are produced, alongside lower levels of the brain chemical BDNF [42]. Low levels of BDNF are associated, in humans, with anxiety and depression. This suggests that a depletion of beneficial bacteria may play a causative role in anxiety and depression. Our dietary intervention sought to repopulate the gut with beneficial bacteria and saw a marked reduction in self-reported feelings of anxiety and depression. There are a number of physiological plausible mechanisms for the way in which gut microbes might influence brain-function by way of the gut-brain axis. It has been found that in germ-free mice (bred to have deficient gut bacteria) there is both an altered stress-response and structural differences in the amygdala and hippocampus–regions implicated in emotion processing and memory [43]. Gut bacteria are also known to have a direct role in the production of serotonin (a neurotransmitter heavily implicated in depression and anxiety), with research demonstrating changes in central nervous system serotonin concentration in germ-free mice [44]. A recent review of probiotic supplementation has suggested a beneficial role for gut bacteria manipulations for alleviating symptoms of depression and anxiety [45].The findings of our current research suggest that dietary manipulations designed to influence gut bacteria may have an important therapeutic role to play in boosting mood in healthy adults and also, potentially, for treating conditions such as anxiety and depression.

RETRACTED

We also identified significant improvements in self-reported cognitive function at the end of the four-week intervention. Participants reported more symptoms on the ‘mind’ sub-scale of the MSQ before undergoing the intervention; these include symptoms such as poor memory and concentration and difficulties making decisions. Interestingly, the dietary protocol of *The Gut Makeover* is very similar to that included in a multi-dimensional therapy used by Bredesen [46,47] for patients in the early stages of Alzheimer’s disease. Alongside exercise and other lifestyle factors, Breseden advocates dietary measures to optimise the microbiome, such as a twelve-hour overnight fast, plentiful vegetables and minimising processed food and grains. Preliminary results, based upon both self-report and neuropsychological testing, suggest improvements in cognitive function for patients with Alzheimer’s disease making these dietary adjustments, as part of a wider protocol. Taken together with our findings, these results suggest that dietary interventions to optimise gut bacteria may have a role to play both in the treatment of Alzheimer’s disease but also in optimising cognitive functioning in non-clinical populations. In their recent review of the evidence of microbiome involvement in Alzheimer’s disease, Hu et al [48] go as far as suggesting that it, ‘may begin in the gut, and is closely related to the imbalance of gut microbiota’. Dietary interventions such as *The Gut Makeover* could be seen as very promising treatment/prevention protocols that warrant further investigation.

This report details an uncontrolled observational study of self-reported symptoms that were recorded within the context of nutritional therapy sessions. As such, there are a number of aspects of methodology that we were not able to control and that need to be borne in mind when interpreting the results. The sample size was relatively small, which would have limited the power to detect a significant change in symptom scores. Despite this, significant reductions in symptoms were noted and there was a marked improvement for each and every participant. It would be important to replicate these findings in a larger sample. The lack of adjustment for confounding variables also impacts upon the reliability of the results. There was no control group in the study and the participants were not blind to the treatment protocol. Therefore, there may have been a significant influence of a ‘placebo-effect’ in producing the dramatic improvements noted. We know that the expectations of participants receiving a therapy can have a dramatic impact on self-reported symptoms. In the treatment of depression, for example, placebo treatments are consistently found to have efficacy rates of 35–40% [49]. For dietary interventions it is much more difficult to conduct the gold-standard placebo-controlled, double-blind studies. However, one factor that suggests that the benefits of the dietary intervention are unlikely to be solely attributable to a placebo-effect, is the large scale improvement in symptoms (such as those related to cognition, emotion and sleep) that were not directly identified as being potential benefits at the outset of the program. For dietary interventions, it is also difficult to monitor adherence to the regime. Given that significant results were observed without being able to control for adherence, we can be fairly confident that the regime is a workable intervention that people can readily follow to a level of compliance that can produce observable benefits. Future research could potentially explore the degree of adherence that is needed to achieve positive results and assess the efficacy of longer-term adherence, by assessing user reported satisfaction. Investigations could also be made into whether any particular aspects of the protocol are more instrumental than others in achieving the positive outcomes. For forthcoming investigations, it will be important to analyse the direct effect of this dietary manipulation on microbiome diversity and health. An increasing number of studies are employing microbial analysis in order to assess the impact of various interventions on gut bacteria and also to explore the impact of gut bacteria on aspects of physiology, including metabolism.[50–52]. By using massive parallel (Next-Generation) high-throughput gene sequencing (as used by ‘Map My Gut’ [53]) we may be able to identify species-specific microbial alteration resulting from the dietary intervention.

RETRACTED

Despite the methodological short-comings of this uncontrolled, observational study, we have uncovered large-scale improvements in physical and emotional well-being and cognitive functioning that are achieved within a four-week time period using this easily implementable dietary intervention. Such rapid, extensive and high-magnitude benefits warrant further detailed investigation using standardised clinical instruments, neuropsychological testing and microbial gene sequencing. The implications of this dietary protocol may be far-reaching. It has the potential for improving physical and emotional wellbeing in the general population and also for being used as part of a treatment protocol for conditions as diverse as IBS, anxiety, depression and Alzheimer’s disease. Given the detrimental side-effects, not to mention limited efficacy, of many medications currently used to treat such conditions, microbiome-focused dietary treatment plans could be seen as a safe and effective first-line therapeutic option.
